# Application Effect of Whole-Process Seamless Nursing Model Based on Smart Healthcare Mode in Perioperative Period of Patients Undergoing Hematoma Removal

**DOI:** 10.1155/2022/1323678

**Published:** 2022-02-23

**Authors:** Chang Liu, Rui Liu, Zhaohua Li, Meiling Tang, Fenghua Wang

**Affiliations:** ^1^Operation Room, the First Affiliated Hospital of Harbin Medical University, Harbin 150001, Heilongjiang, China; ^2^Library Room, Harbin Children's Hospital, Harbin 150000, Heilongjiang, China; ^3^Department of Medical Section, the First Affiliated Hospital of Harbin Medical University, Harbin 150001, Heilongjiang, China

## Abstract

**Objective:**

To explore the application effect of a whole-process seamless nursing model based on the smart healthcare mode in the perioperative period of patients undergoing hematoma removal.

**Methods:**

In this retrospective study, 50 patients with hematoma removal admitted to our hospital from August 2018 to August 2019 were included as the control group (CG), while 50 patients with hematoma removal admitted to our hospital from September 2019 to September 2020 were included as the experimental group (EG). During the period of hematoma removal, CG received routine perioperative nursing, while EG received the whole-process seamless nursing model based on the smart healthcare mode. The perioperative indexes, hemodynamic indexes, and the incidence of postoperative complications were compared between the two groups, and the incidence of nursing staff's work omissions in different periods was analyzed.

**Results:**

Notable differences were observed in surgical time, intraoperative blood loss, hematoma clearance rates, length of ICU stay, hospitalization time, removal time of ventricular drainage tube, and cerebral edema volume at 1 week after surgery between EG and CG (*P* < 0.05). Compared with CG, EG achieved obviously better hemodynamic indexes (*P* < 0.001) and a lower incidence of bedsore, muscle atrophy, and eating/swallowing disorders (*P* < 0.05). During the implementation of smart healthcare, the incidence of nursing staff's work omissions was remarkably reduced (*P* < 0.05).

**Conclusion:**

Under the smart healthcare, the incidence of nursing staff's work omissions is lower, and the effect of the whole-process seamless nursing is better, which can optimize the perioperative indexes of patients, stabilize the postoperative hemodynamics, and reduce the incidence of complications. Therefore, the whole-process seamless nursing model based on the smart healthcare mode has promotion value in clinic.

## 1. Introduction

Intracranial hematoma, the most common secondary lesion of craniocerebral injury, is often caused by abnormal accumulation of intracranial hemorrhage in the cranial cavity. The disease will cause increased intracranial pressure and brain tissue damage in patients, subsequently triggering a series of clinical symptoms such as disturbance of consciousness and memory decline. Without timely intervention, patients may suffer from complications such as cerebral ischemia and irreversible neurological dysfunction, which seriously endanger their life and health [1, 2]. At present, its clinical treatments mainly include conservative treatment and surgical treatment, in which only surgical treatment can eliminate hematoma. Therefore, patients meeting the surgical indications without surgical contraindications should receive surgical treatment as soon as possible. In particular, hematoma removal should be performed in patients with severe craniocerebral injury to reduce the risk of death [3, 4].

Though hematoma removal can quickly remove the hematoma, alleviate the occupying effect, and reduce the pressure of hematoma on normal brain tissues, it puts forward higher requirements for nursing, and its combination with high-quality perioperative nursing can minimize the potential tissue damage and improve surgical outcomes. Camicia Michelle et al. have reported that seamless nursing is able to enhance the continuity of perioperative nursing and reduce patients' psychological pressure on surgery [5]. Some studies have applied it in hematoma removal and found that this nursing model reduces the incidence of postoperative complications such as postoperative pulmonary infection and muscular atrophy, improves the nursing satisfaction of patients, and reduces nurse-patient disputes [6, 7]. In recent years, with the further promotion of the smart healthcare, many hospitals have developed an integrated platform of nursing information to share online medical resources and effectively solve the problem of difficult integration of nursing information among various systems. The data sharing and objectivity of smart healthcare bring more possibilities to the seamless nursing because the online platform can optimize the operation process, improve the nursing efficiency, and effectively reduce the possibility of nursing omissions [8, 9]. On the basis of routine nursing assisted by smart healthcare platform, nursing staff only need to adopt the evidence-based nursing to gradually improve the seamless nursing model and deepen the nursing details, thereby comprehensively enhancing the service quality. At present, there is no research on smart healthcare platform as the basis of seamless nursing. Based on this, this paper combined the two in patients with hematoma removal to further improve the perioperative nursing effect.

## 2. Materials and Methods

### 2.1. Study Design

This retrospective study was conducted in our hospital from August 2018 to September 2020 to explore the application effect of a whole-process seamless nursing model based on the smart healthcare mode in the perioperative period of patients undergoing hematoma removal.

### 2.2. Inclusion Criteria and Exclusion Criteria

Inclusion criteria: (1) patients were confirmed with intracranial hematoma by head CT or MRI and underwent hematoma removal [10]; (2) patients are aged no less than 18 years old; (3) the time from onset to treatment of the patients was within 24 hours; and (4) patients were treated in our hospital throughout the whole process and had complete clinical data.

Exclusion criteria: (1) patients had severe organic diseases; (2) patients had mental illness or other factors affecting communication; (3) patients did not pass the drug sensitivity test; (4) patients had seriously abnormal coagulation function or took anticoagulants and antiplatelet drugs within one week after the onset; and (5) patients were in pregnancy or lactation.

### 2.3. General Data of Patients

Fifty patients with hematoma removal admitted to our hospital from August 2018 to August 2019 were included as the control group (CG), while 50 patients with hematoma removal admitted to our hospital from September 2019 to September 2020 were included as the experimental group (EG). No notable differences in general data were found between the two groups (*P* > 0.05), see Section 2.1.

### 2.4. Ethical Consideration

This study was in line with the principles of Helsinki Declaration (2013) [11]. After the patients were recruited, the research group explained the study purpose, significance, content, and confidentiality to them and asked them to sign the informed consent.

### 2.5. Methods

The CG patients received routine perioperative nursing. Before surgery, the nursing staff performed preoperative education, carefully checked the patients' surgical information, and prepared the surgical instruments and drugs. During surgery, the staff closely monitored the patients' physical data such as heart rate, blood oxygen saturation, blood pressure, and body temperature and cooperated with the doctors to help patients maintain the appropriate position and protect their privacy. After surgery, the staff helped to wipe the blood on the patients, sent them to the wards, and did the handover. Then, the nursing staff in the wards closely observed the changes of patients' condition and signs.

The EG patients group received the whole-process seamless nursing model based on the smart healthcare mode, with the following measures based on the routine nursing in CG. (1) A seamless nursing group was established, including a senior and experienced nursing staff as the leader, a nursing staff with strong communication ability as the deputy leader, the head nurse of the department as the counselor, 20 nursing staff with professional training and specialist work experience over 3 years as the team members, and 2 nursing staff as the office staff. Through evidence-based nursing, team members consulted relevant guidelines and literature, consulted the experts, listened to related lectures, and cultivated awareness of smart healthcare. (2) The seamless nursing group and the R&D personnel of the software development company jointly established the smart healthcare management platform, including four systems. One was the nursing workstation system, mainly including medical advice processing module, surgery appointment module, and medical instrument management module. The nursing staff accessed and operated the platform through the mobile client. The second one was laboratory and inspection configuration system. The office nursing staff generated project labels through computer operation after checking the medical orders of test or inspection in the medical advice processing module and arranged the patients for examination. The third was nursing information management system, including nursing electronic medical records, nursing quality control, head nurse scheduling, adverse event reporting, and nursing safety monitoring. The fourth was the electronic display board system. The nursing staff consulted patient information, shift information, patient vital sign monitoring data, catheter data, nursing assessment, relevant doctor's advice, nursing records, and test and examination results on the electronic display board. The above data were updated in real time, the nursing staff could modify the data on any interface, and the office nursing staff were responsible for checking. (3) The seamless nursing group logged into the smart healthcare management platform and reviewed and processed the patients' medical orders (nursing level, diet, laboratory test, and examination). Operated online by office nursing staff without manual entry and transcription, the platform automatically printed the orders into treatment sheets, infusion sheets, injection sheets, and appointment numbers. The perioperative nursing measures in the standardized process of seamless nursing for hematoma removal were directly generated by the smart healthcare system. (4) On the basis of routine nursing measures issued by the smart healthcare system, combined with the nursing risks in the operating room and the actual situation of patients with hematoma removal over the years, the group summarized the problems existing in the perioperative nursing, and then formulated a more detailed seamless nursing scheme, mainly including preoperative visits, intraoperative nursing and postoperative nursing. (5) Before surgery, the nursing staff performed health education to patients to alleviate their negative psychological state and help them to overcome fear. During surgery, the staff strictly controlled the temperature and humidity in the operating room and massaged the patients' limbs to promote blood circulation for those with long surgical time. After surgery, the staff did handover, helped patients wake up as soon as possible, wear clothes and cover the quilt, and fixed the drainage tube. After recovery, the staff visited the patients again to inform them of the possible postoperative complications and precautions and provided psychological comfort for them.

### 2.6. Observation Criteria

General data: after the patients were enrolled, the general data were collected, and the information files were established, including gender, age, height, weight, BMI, Glasgow Coma Scale (GCS) index [12], and hematoma volume.

Perioperative indexes: perioperative indexes included surgical time, intraoperative blood loss, hematoma clearance rate, length of ICU stay, hospitalization time, removal time of ventricular drainage tube, and cerebral edema volume at 1 week after surgery.

Hemodynamic indexes: electrocardiogram (TLC6000, Hebei Medical Products Administration certified No. 20102210047) was performed to monitor the patients' heart rate at 1 day before surgery and 1 day after surgery. The standard mercury sphygmomanometer (Jiangsu Yuwell Medical Equipment Co, Ltd.; Jiangsu Medical Products Administration certified no. 20152070945) was adopted to monitor the patients' blood pressure at 1 day before surgery and 1 day after surgery and to calculate the mean arterial pressure (MAP).

Incidence of postoperative complications: the complications included bedsore, muscle atrophy, pulmonary infection, eating/swallowing disorders, hypostatic pneumonia, acute ulcer hemorrhage of digestive tract, and joint stiffness. The number of patients with complications was recorded.

Incidence of work omissions: the 24 nursing staff's work omissions from August 2018 to August 2019 and from September 2019 to September 2020 were recorded, including transcribe errors of infusion sheets, transcribe errors of doctor's advice, errors or omissions of infusion sheets, errors or omissions of laboratory labels, information errors of electronic display board, and nurse-patient disputes.

### 2.7. Statistical Treatment

The data in this study were processed by the SPSS20.0 software and graphed by GraphPad Prism 7 (GraphPad Software, San Diego, USA). This study included enumeration data and measurement data, tested by X^2^ and *t*-test. The differences were statistically significant at *P* < 0.05.

## 3. Results

### 3.1. General Data

The EG had 30 males and 20 females, with an average age of 44.02 ± 16.86 years old, average height of 172.65 ± 15.11 cm, average body weight of 60.98 ± 5.65 kg, average BMI of 22.65 ± 2.32 kg/m^2^, average GCS score of 7.22 ± 1.10, and average hematoma volume of 50.22 ± 10.26 mL. CG had 28 males and 22 females, with an average age of 43.96 ± 17.42 years old, average height of 172.78 ± 15.23 cm, average body weight of 61.18 ± 5.60 kg, average BMI of 22.41 ± 2.30 kg/m^2^, average GCS of 7.25 ± 1.10, and average hematoma volume of 50.12 ± 10.28 ml. No notable differences in general data were found between the two groups (*P* > 0.05).

### 3.2. Perioperative Indexes

Notable differences in the perioperative indexes were observed between EG and CG (*P* < 0.05), see Table 1.

### 3.3. Hemodynamic Indexes

The postoperative hemodynamic indexes were notably better in EG than in CG (*P* < 0.001), as presented in Figure 1.

No notable differences in heart rates and MAP were observed between EG and CG at 1 day before surgery (69.23 ± 2.65 vs. 69.50 ± 2.44 and 85.65 ± 5.20 vs. 87.00 ± 5.23; *P* > 0.05). The heart rate and MAP in EG were obviously lower than those in CG at 1 day after surgery (72.11 ± 2.65 vs. 78.65 ± 2.68 and 89.68 ± 5.65 vs. 95.11 ± 5.47; *P* < 0.001).

### 3.4. Incidence of Postoperative Complications

The incidence of bedsore, muscular atrophy, and eating/swallowing disorders in EG was remarkably lower compared with CG (*P* < 0.05), see Table 2.

### 3.5. Incidence of Work Omissions

During the implementation of smart healthcare, the incidence of nursing staff's work omissions was remarkably reduced (*P* < 0.05), as presented in Table 3.

## 4. Discussion

Intracranial hematoma is the abnormal blood aggregation caused by vascular rupture between brain or brain tissues and skull. The disease includes acute intracranial hematoma and spontaneous intracranial hemorrhage, in which the former is caused by skull deformation and fractures after traumas and the latter is caused by diseases such as hypertension and cerebrovascular diseases [13, 14]. The manifestations vary in the different types of hematoma, but most patients have varying degrees of consciousness disorder and a small number of patients are complicated with symptoms such as mental retardation and memory decline, which should be timely treated according to the different conditions of patients. For patients with less blood loss and mild craniocerebral injury, conservative treatment is generally adopted. For patients with supratentorial hemorrhage above 30 mL, subtentorial hemorrhage above 10 mL or with cerebral hernia, hematoma removal should be performed immediately [15–17]. Hematoma removal is an important measure to reduce the changes of secondary diseases, with high requirements for nursing. Therefore, excellent perioperative nursing can effectively improve the surgical indicators of patients and boost the therapeutic effect [18]. At present, some scholars have applied seamless nursing in patients with hypertension undergoing craniotomy hematoma removal and achieved excellent results in reducing postoperative complications and improving the nurse-patient relationship. With the people-oriented nursing concept throughout the whole process, this nursing model aims to provide complete and continuous nursing services for patients. Additionally, the nursing staff need to constantly find problems and defects in the nursing process and then make modifications, thereby improving the nursing quality and eliminating the disadvantages of nursing services. The study of Xiao Feina and others has shown that seamless nursing improves the perioperative indexes of patients, with an average surgical time of 80.61 ± 10.54 min [19]. This study also achieved the same results, indicating that seamless nursing has exact value in the perioperative nursing of patients undergoing hematoma removal. However, the seamless nursing model is rarely applied in practice, and its application is subject to various factors, among which the most critical factor lies in the cooperative work of nursing staff and the sharing of nursing information. Without high-speed and accurate intercommunication of medical resources, seamless nursing cannot play its practical role.

In recent years, the development of smart healthcare has provided more possibilities for the application of seamless nursing. Characterized by digitalization, automation, and intelligence, the smart healthcare management platform can standardize the nursing information system and simplify the nursing management process, especially avoiding the potential safety hazards caused by human factors in nursing work and shortening the handover time of nursing staff [20–22]. The application of smart healthcare management in seamless nursing can effectively improve the efficiency of collaborative work among nursing staff and increase the timeliness and scientificity of nursing work. With the support of this kind of information technology, nursing staff have fewer work omissions [23, 24]. Therefore, the incidence of work omissions during the implementation of smart healthcare mode was significantly reduced (*P* < 0.05). Since the smart healthcare system has issued a routine process of seamless nursing, the workload of nursing staff is greatly reduced. The nursing staff can spend more time on the evidence-based nursing, learn from previous nursing, optimize seamless nursing measures, and provide patients with comprehensive and high-quality nursing [25]. Therefore, the patients in EG had more stable physical indicators after surgery and a lower incidence of bedsore, muscle atrophy and eating/swallowing disorders, suggesting that smart healthcare is a good basis for seamless nursing and can improve the application effect of this nursing model.

Hematoma removal is an important way to treat intracranial hematoma. Under the smart healthcare, the incidence of nursing staff's work omissions is lower, and the effect of the whole-process seamless nursing is better, which can optimize the perioperative indexes of patients, stabilize the postoperative hemodynamics, and reduce the incidence of complications. Therefore, the whole-process seamless nursing model based on the smart healthcare mode has promotion value in clinic.

## Figures and Tables

**Figure 1:** Comparison of patients' hemodynamic indexes (‾*x* ± *s*). Note: the abscissa of Figures 1(a) and 1(b) from left to right represented 1 day before and 1 day after surgery. The black area denotes EG, while the gray area denotes CG. # indicates *P* < 0.001.

**Table 1:** Comparison of patients' perioperative indexes.

Group	EG (*n* = 50)	CG (n = 50)	X^2^/*t*	*P*
Surgical time (min)	78.65 ± 10.22	123.32 ± 15.32	17.152	<0.001
Intraoperative blood loss (mL)	44.21 ± 5.65	154.98 ± 13.65	53.019	<0.001
Hematoma clearance rate (%)	96.0(48/50)	84.0(42/50)	4.000	0.046
Length of ICU stay (d)	2.67 ± 0.54	3.10 ± 0.35	4.725	<0.001
Hospitalization time (d)	7.32 ± 1.51	9.24 ± 1.23	6.971	<0.001
Removal time of ventricular drainage tube (d)	3.44 ± 0.84	4.96 ± 0.65	10.119	<0.001
Cerebral edema volume at 1 week after surgery (mL)	24.12 ± 2.55	28.65 ± 2.10	9.697	<0.001

**Table 2:** Comparison of the incidence of postoperative complications (*n*(%)).

Group	EG (*n* = 50)	CG (*n* = 50)	X^2^	*P*
Bedsore	0(0.0)	4(8.0)	4.167	0.041
Muscle atrophy	0(0.0)	4(8.0)	4.167	0.041
Pulmonary infection	1(2.0)	3(6.0)	1.042	0.307
Eating/swallowing disorders	0(0.0)	4(8.0)	4.167	0.041
Hypostatic pneumonia	0(0.0)	3(6.0)	3.093	0.079
Acute ulcer hemorrhage of digestive tract	0(0.0)	3(6.0)	3.093	0.079
Joint stiffness	1(2.0)	5(10.0)	2.837	0.092

**Table 3:** Comparison of the incidence of nursing staff's work omissions in different periods [n(%)].

Group	September 2019 to September 2020 (*n* = 24)	August 2018 to August 2019 (*n* = 24)	X^2^	*P*
Transcribe errors of infusion sheets	0(0.0)	1(4.2)	1.021	0.312
Transcribe errors of doctor's advice	1(4.2)	2(8.3)	0.356	0.551
Errors or omissions of infusion sheets	0(4.0)	2(8.3)	2.087	0.149
Errors or omissions of laboratory labels	1(4.2)	2(8.3)	0.356	0.551
Information errors of electronic display board	0(0.0)	3(12.5)	3.200	0.074
Nurse-patient disputes	0(0.0)	2(8.3)	2.087	0.149
No omissions	23(95.8)	18(75.0)	4.181	0.041

## Data Availability

Data to support the findings of this study are available on reasonable request from the corresponding author.
